The article "Study of Fano Resonance Effects in Graphene-Grating Composite Structures" was published in 2022. Journal: Comput Intell Neurosci.

# Study of Fano Resonance Effects in Graphene-Grating Composite Structures

**DOI:** 10.1155/2022/8446093

**Published:** 2022-09-01

**Authors:** Danying Cui, Jin Liu, Haima Yang

**Affiliations:** ^1^School of Electronic and Electrical Engineering, Shanghai University of Engineering Science, Shanghai 201620, China; ^2^School of Optical-Electrical and Computer Engineering, University of Shanghai for Science and Technology, Shanghai 200093, China

## Abstract

In order to optimize the sensitivity and detection accuracy of Fano resonance optical sensors, a sensing model of graphene-grating composite micro-nanostructure with high sensing performance is proposed based on the optical properties of graphene and grating. By studying the reflection spectra and field distribution characteristics of the structure, the sensing mechanism of Fano resonance generated by the structure is elaborated, and the parameters affecting the Fano resonance sensing performance are analyzed to enhance the Fano resonance sensing performance by optimizing the structural parameters, and the Fano resonance reflection spectral curve with high-sensitivity and high-quality factor (FOM) value is obtained. The results show that when the grating period *P*=300 nm, the grating height *T*1 = 110 nm, and the silver film thickness *T*2 = 30 nm, the sensitivity of the structure is 980 nm/RIU and the quality factor FOM is 770RIU^−1^ by changing the refractive index of the material to be measured.

## 1. Introduction

Fano resonance has received increasing attention in recent years with the development of nanophotonics. Fano resonance sensing is a contamination-free, marker-free, real-time detection optical sensing technique that is usually excited by light waves incident on the sensor surface [1]. In contrast to the Lorentzian resonance line pattern, which exhibits symmetrical resonance line pattern within the spectrum, the Fano resonance line pattern, which exhibits asymmetrical resonance line pattern, is induced by phase extinction interference between light in the continuous state and light in the discrete state under specific phase-matching conditions and is mainly characterized by its ability to change rapidly in a narrow wavelength range [2]. Therefore, optoelectronic devices designed based on Fano resonance have the advantages of short response time, low loss, and high sensitivity, making them more practical. Such optoelectronic devices have been widely used in many fields, including refractive index sensors [3, 4], biosensors [5, 6], and medical diagnostics [7, 8]. Optimization of Fano sensor parameters to improve sensitivity and detection accuracy has become a major research challenge. In nanophotonics, grating structures are often used to achieve Fano resonance, which is due to the ability of grating structures to combine with various dielectric or metallic materials to more easily excite narrower resonance peak spectral curves and thus obtain higher sensitivity [9, 10]. Zheng et al. [11] proposed a tunable resonant two-sided dielectric grating structure, which uses a vertically incident plane wave to excite. The maximum electric field intensity in the grating spacer layer of this structure was increased by a factor of 35 compared to the incident field, and the sensitivity reached 602.15 nm/RIU. Wang et al. [12]proposed grating-coupled micro and nanosensing structures consisting of several layers of graphene and a germanium prism with a multilayer film, using the graphene surface of the graphene-dielectric interface to equipartition. The interaction between the excitation mode and the planar waveguide mode formed an asymmetric Fano resonance line shape in the spectrum, and the measured material was introduced into the structure with a sensitivity up to 681 nm/RIU. Wen et al. [13] designed a refractive index sensing structure based on an all-grating resonant cavity, which achieves Fano resonance through the mutual coupling of two subwavelength grating track resonators. The structure has a maximum sensitivity of 500 nm/RIU. Chen et al. [14] proposed a hybrid structure of a subwavelength grating all-dielectric multilayer film containing a periodic photonic crystal, which formed a Fano resonance by coupling the discrete states generated by the subwavelength waveguide grating with the continuous states generated by the photonic crystal cavity, and obtained the sensing characteristics with high FOM value. Lo et al. [15] proposed a nanoslit grating array structure covered by aluminum metal, which utilizes the coupling of the aluminum film and grating structure to achieve asymmetric Fano resonance, and its sensitivity can reach 470 nm/RIU. At present, the micro-nanostructures based on Fano resonance mostly focus on the novelty of the structural design, but the preparation of the structure requires high process requirements, and few metal grating structures with simple rectangular profiles are introduced in two-dimensional super materials. There are few reports on the introduction of two-dimensional super materials into the metal grating structures with simple rectangular profiles to enhance the sensing characteristics of Fano resonance.

In this paper, a composite micro-nanograting structure with the introduction of graphene is proposed. The structure deposits a layer of graphene on top of a three-layer Au-Ag-SiO_2_ nanograting structure, and under the condition of wave vector matching, the reflected signal in the graphene-Au grating structure is used as a discrete optical signal to interfere with the discrete optical signal generated in the metal Ag film of the dielectric layer in the nanograting structure to excite Fano resonance in the structure.

We first construct a Fano resonance sensing structure model based on wavelength modulation, analyze the sensing mechanism of generating Fano resonance, and then analyze the effects of different structural parameters on the sensing characteristics by using the time-domain finite difference method, and at the same time, we carry out parameter optimization to obtain a sensing structure model with good performance.

## 2. Structural Modeling and Theoretical Analysis

### 2.1. Model Structure Construction

In this paper, a graphene-grating composite micro-nanostructure sensing model is proposed, and the geometric model is established by using the time-domain finite difference analysis software FDTD solutions [16–20], as shown in Figure 1. The Au grating with period P and depth T1 is placed on the metal Ag film with thickness T2. The graphene layer is coated on the Au nanograting, the sensing medium is fixed on the top of the grating, the dielectric layer of the structure is selected from the metal Ag film with thickness T2, the substrate is selected from the SiO_2_ with thickness T2, and the incident light is incident at an angle *θ*, which constitutes the whole parameter system. Deionized water with a refractive index of 1.333 is now used as the test object, and the initial parameters of the graphene-grating sensing model are set as follows: *P* =300nm, *T*_1_ =70nm, *T*_2_ =10nm, *T*_3_ =600nm, and *θ*=0°, and the Fano resonance is excited with the planar light of TM mode as the incident light. The simulation is performed with one grating period as a cell in the *X*-direction, and a perfectly matched layer (PML) is added as an absorption boundary condition in the *Y*-direction. In this paper, a plane wave light source of 450–600 nm is used to analyze its optical sensing characteristics under wavelength modulation in detail.

The graphene coating on the Au grating in this structure can make the energy more localized and prevent the metal from oxidation [21–25]. In addition, the dielectric constant of graphene has many similarities with metals, and when the imaginary part of the conductivity of graphene is greater than zero, the surface equipartition excitations in TM mode will be excited by the metallic nature exhibited by graphene and produce a strong field localization effect. The electrical conductivity of graphene can be expressed according to the Drude model as

(1) $$\begin{array}{c} \sigma_{\text{g}}=\frac{e^{2}E_{\text{f}}}{\pi \hbar^{2}}\frac{i}{\omega +i\tau^{-1}}, \end{array}$$

where *e* is the meta-charge, *E*_f_ is the Fermi energy level of graphene, *ℏ* is Planck's constant, *ω* is the incident light angular frequency, *τ* is the carrier relaxation time, and *μ* is the carrier mobility.

### 2.2. Theoretical Analysis

Surface plasmon polaritons (SPPs) are highly localized electromagnetic waves that propagate along the surface of a dielectric and a metal. The electric field intensity is maximized at the metal-dielectric interface and is confined and decays exponentially in the vertical direction of the metal surface [26–33]. When the surface equipolar excitations are excited, there is an energy transfer from the incident light to the surface equipolar excitations, which reduces the intensity of the reflected light. In the case of incident TM polarized light, the dispersion relation of surface equiaxed excitations transmitted by SPPs along the dielectric metal-intersection is

(2) $$\begin{array}{c} k_{SPPs}=k_{0}\sqrt{\varepsilon_{g}\varepsilon_{m}/\left(\varepsilon_{g}+\varepsilon_{m}\right)}, \end{array}$$

where *k*_0_ is the incident light wave vector, *ε*_g_ is the dielectric constant of graphene, and *ε*_m_ is the dielectric constant of the dielectric grating.

At the same frequency, the incident light wave vector *k*_0_ is always smaller than the wave vector *k*_*SPPs*_ of the surface equipartition excitations, resulting in the inability to match *k*_*SPPs*_ with *k*_0_. In order to be able to excite SPPs, special optical structures are needed to match the incident light wave vector with the wave vector of the surface plasmon polaritons. SPPs are excited by prism coupling excitation, waveguide coupling excitation, fiber coupling excitation, and grating coupling excitation. In the grating coupling technique, the horizontal tangential component of the wave vector is

(3) $$\begin{array}{c} k_{x}=k_{0}n_{a}\sin\theta \pm m\left(\frac{2\pi }{P}\right), \end{array}$$

where $n_{a}=\sqrt{\varepsilon_{a}}$ is the refractive index of the dielectric located at the grating notch, *θ* is the resonant incidence angle of the SPPs, *m* is the diffraction level of the dielectric grating, and *P* is the grating period.

When *k*_*x*_=*k*_*SPPs*_ is compensated by the grating diffraction effect, *k*_0_ can be matched with *k*_*SPPs*_, which makes the SPPs excited. At this time, the resonance wavelength *λ* = 489 nm, and the electric field distribution of the SPPs generated in the graphene-grating structure are shown in Figure 2(b). It can be seen that a large amount of electromagnetic field energy is localized near graphene, and the electric field energy distribution decays gradually in the vertical direction, which is consistent with the theory of SPPs. After the incident light achieves wave vector matching in the graphene-grating structure, the reflected light energy decreases sharply, which indicates that after the incident light resonates in the graphene-grating structure, most of the energy is absorbed by graphene. Thus, in the case of resonance, the majority of the incident light will be consumed and cannot return to the incident medium again, making the reflected light energy decrease sharply, thus forming the narrow-band shown in Figure 2(a) peak, the discrete state required for the Fano resonance. However, a very small amount of energy also penetrates through the graphene layer to reach the dielectric layer metal Ag film, thus forming a wider band in the reflection spectral curve and providing a continuous state for the Fano resonance with stable optical effects, as shown in the continuous state spectral curve in Figure 2(a). Among them, the graphene-grating structure provides the discrete state by generating SPPs, and the lower dielectric layer metal Ag film provides the continuous state by generating a broadband band. Under the condition of satisfying the wave vector matching, the discrete state curve will be redshifted or blueshifted in a certain wavelength range along with the change of the environmental parameters to be measured and then coupled with the same frequency components in the continuous state to make the reflection spectral line shape change dramatically. The process of Fano resonance realization is shown in Figure 2(a).

## 3. Results and Discussion

In order to achieve the best performance of the designed structure, the relevant structural parameters need to be optimized and analyzed. The reflection spectrum is analyzed by varying the individual structural parameters to find the optimum performance of the sensor, and the optimization of the sensor structural parameters is finally completed. In this paper, using wavelength modulation, one of the performance parameters of the sensor, sensitivity S, refers to the sensitivity of the detected variable to changes in refractive index, and sensitivity S can be expressed as

(4) $$\begin{array}{c} S=\frac{\Delta \lambda }{\Delta n_{\text{d}}}, \end{array}$$

that is, the ratio between the amount of change in the resonance wavelength and the amount of change in the refractive index of the medium.

Full width at half maximum (FWHM) is also an evaluation index of the sensor, indicating the width of the incident light wavelength when the resonance depth reaches half, and the narrower the FWHM of the resonance peak, the higher the resolution and the smaller the sensor loss.

The depth of resonance (depth) is the height of the resonance peak in the reflection spectrum, which can indicate the coupling efficiency of energy. The greater the depth of resonance, the higher the coupling efficiency between the surface plasma wave and the incident light wave.

The quality factor FOM value can be evaluated by the resonance peak shape of the spectrum to evaluate the performance of the sensor and is equal to the ratio of the sensitivity S to the full width at half peak FWHM of the resonance curve.

The definition of quality factor is proposed:

(5) $$\begin{array}{c} \text{FOM}=\frac{S}{\text{FWHM}}. \end{array}$$

As can be seen from (5), when S is larger, the smaller the FWHM, the larger the FOM, which indicates that the better the performance of the sensor, and vice versa, the worse the performance of the sensor.

### 3.1. Effect of Grid Height H on Sensing Characteristics

The grating structure is an important component of the overall sensor, so the parameters of the grating structure can have a significant impact on the sensor performance. The grating height H values are set to 70 nm, 80 nm, 90 nm, 100 nm, and 110 nm for simulation, and the results obtained from the simulation are shown in Figure 3(a). It can be seen that the structure produces good Fano resonance properties, and the resonance curve gradually redshifts with increasing grating height, with a slight increase in the peak reflectivity, indicating that the increase in grating height makes its ability to localize photons enhanced. The resonant peak depth and full width at half maximum (FWHM) do not vary significantly, but the resonant peak depth is more influenced by the grating height compared to FWHM, and the trend of resonant peak depth with grating height is shown in Figure 3(b). It can be seen from the figure that when the grating height is 110 nm, the peak depth of the resonance is greater, which means that the Fano resonance coupling intensity is greater at this time, thus leading to enhanced interference between the grating and the graphene structure, so the grating height of 110 nm is chosen to continue the analysis.

### 3.2. Effect of the Grating Period P on Sensing Characteristics

When TM polarized light is incident, the medium grating equivalent refractive index can be expressed by the following expression:

(6) $$\begin{array}{c} n_{0,TM}=\frac{n_{H}n_{L}}{{\left[fn_{L}^{2}+\left(1-f\right)n_{H}^{2}\right]}^{1/2}}, \end{array}$$

where *n*_*H*_ and *n*_*L*_ correspond to the high and low refractive index of the dielectric grating, and *f*=*l*/*P* is the duty cycle of the grating structure, where *l* is the ridge width of the dielectric grating.

From (3) and (6), it can be seen that the wave vector matching condition and the equivalent refractive index will be affected by the grating period, and the regulation of SPPs in the graphene/grating/dielectric layer structure can be accomplished by changing the grating period to achieve the optimization of the reflection spectral curve and sensing performance of the structure. Under the condition of grating height *H* = 110 nm, the grating period P is adjusted and the grating periods are set to 300 nm, 325 nm, 350 nm, 375 nm, and 400 nm for simulation, and the reflection spectra shown in Figure 4(a) are obtained. It can be observed that the resonance intensity and position of the reflection spectrum change significantly with the change of grating period, and the peak of the reflection spectrum curve decreases and then increases. As shown in Figure 4(b), the change of resonance depth is with the change of the grating period. It can be seen that the resonance depth decreases and then increases with the increase of the grating period, and the resonance depth is maximum when the grating period is 300 nm, which means that the coupling strength between the structures is maximum at this time. Therefore, the grating period *P*=300 nm is chosen as the optimal value for this sensor, so as to obtain higher sensitivity. The comparison of the depth of the electric field energy color shows that the electric field energy is enhanced with the increasing grating period, which is consistent with the trend of the reflection curve.

### 3.3. Effect of Metal Ag Film Thickness of Dielectric Layer on Sensing Characteristics

At a fixed angle of incidence, the thickness of the metal-dielectric layer directly affects the degree of coupling between the continuous and discrete states. Under the condition that the grating height *H* = 110 nm and the grating period *P*=300 nm remain unchanged, the thickness T2 of the metal Ag film is adjusted to complete the optimization of the sensing characteristics of the structure and the reflection spectrum curve. The thickness of the silver film was set to be 10 nm, 15 nm, 20 nm, 25 nm, and 30 nm, respectively, and the simulation was performed, and the reflection spectrum shown in Figure 5(a) was obtained. As the thickness of the metal Ag film increases, the reflectance spectrum also changes accordingly. It can be seen that the reflectivity in the graphene-grating structure increases with the increase of the thickness of the metal Ag film, which indicates that the graphene-grating structure increases continuously. The coupling efficiency between the structure and the metal Ag thin film of the dielectric layer is also continuously improved. Figure 5(b) shows a partial enlarged view of the resonance peak. It can be seen from the figure that when the thickness of the silver film increases from 10 nm, the full width at half maximum FWHM of the reflection spectrum curve gradually becomes larger, and the resonance depth gradually deepens, indicating that the thickness of the silver film has an effect on the Fano resonance. The degree of loss has a certain impact, but the overall change is not obvious. The resonance peak of the reflection spectrum has changed significantly; as shown in Figure 5(c), the fitting curve between the thickness of the metal Ag thin film and the resonance peak shows a good linear relationship. It can be seen from the figure that when the thickness of the silver film is 30 nm, the resonance peak is the largest, which indicates that the coupling efficiency of Fano resonance reaches the highest at this time, so *d*_A_ = 30 nm is selected as the optimal value of the sensor.

Based on the above analysis, the optimized sensor structure parameters are finally determined as grating height *H* = 110 nm, grating period *P*=300 nm, and silver film thickness *d*_A_ = 30 nm. Then, analyze the sensing characteristics of the optimized structure and set substances to be tested with different refractive indices to observe the shift of the resonance wavelength, so as to obtain the sensitivity of the structure. The medium refractive index of the substance to be measured is set as 1.333, 1.335, 1.337, 1.339, and 1.341, respectively, and the reflection spectrum is obtained as shown in Figure 6(a). It can be seen that the reflection spectrum curve of the structure has a red shift with the increase of the refractive index of the medium to be tested, and the relationship between the refractive index of the tested object and the resonance wavelength is approximately linear. The structure is at 511.4 nm, 513.3 nm, Fano resonance occurs near 516.3 nm, 517.8 nm, and 519.4 nm, and the accuracy of the refractive index change of the object to be measured reaches the order of 10^−3^. The change of the resonance wavelength with the refractive index is shown in Figure 6(b), and the slope of the obtained straight line is the sensitivity (Δ*λ*/Δ*n*) of the sensor. The calculation shows that the value of the sensitivity is 980 nm/RIU. The FOM value of the sensor under different refractive indices is calculated by the formula of the quality factor FOM value, as shown in Figure 6(c), where the maximum FOM value is 770RIU^−1^. It can be seen that the performance of the sensor will also increase with the increase in the refractive index of the material.

## 4. Conclusion

A graphene-grating composite micro-nanosensing structure based on wavelength modulation is proposed. The incident light passes through the graphene-grating structure to generate SPPs to provide discrete states of a narrow-band single frequency. Broadband continuous state, discrete state, and continuous state are coupled under the condition of wave vector matching, thus forming Fano resonance. The sensing characteristics of the structure are analyzed by the time-domain finite difference method. The results show that when the grating height is *T*1 = 110 nm, the grating period *P*=300 nm, and the thickness of the metal Ag film in the dielectric layer is *T*2 = 30 nm, the structure exhibits relatively high performance. Good sensing performance, its sensitivity is 980 nm/RIU, and the quality factor FOM value is as high as 770RIU^−1^. The results of this paper provide new ideas and methods for designing Fano micro-nanosensing structures with simple processes.

## Figures and Tables

**Figure 1:** Schematic diagram of graphene-grating structure sensing.

**Figure 2:** Reflection spectrum and electric field distribution. (a) Reflection spectrum. (b) Electric field map.

**Figure 3:** (a) Reflection spectra of different grating heights. (b) Variation of formant depth with grating height.

**Figure 4:** (a) Reflection spectra of different grating periods. (b) Variation of formant depth with the grating period.

**Figure 5:** (a) Comparison of reflection spectra of different silver film thicknesses. (b) Enlarged formant. (c) Variation of resonance peak with silver film thickness.

**Figure 6:** (a) Reflection spectra of different refractive indices. (b) The relationship between resonance wavelength and refractive index. (c) FOM value under different refractive indices of the object to be measured.

## Data Availability

The data used to support this study are available from the corresponding author upon request.

## References

[1] Gao W., Hu X., Li C. (2018). Fano-resonance in one-dimensional topological photonic crystal heterostructure. *Optics Express*.

[2] Limonov M. F., Rybin M. V., Poddubny A. N., Kivshar Y. S. (2017). Fano resonances in photonics. *Nature Photonics*.

[3] Liu H. G., Zheng L., Ma P. Z. (2019). Metasurface generated polarization insensitive Fano resonance for high-performance refractive index sensing. *Optics Express*.

[4] Wang Z., Fu Z. Y., Sun F., Wang C., Zhou J., Tian H. (2019). Simultaneous sensing of refractive index and temperature based on a three-cavity-coupling photonic crystal sensor. *Optics Express*.

[5] Li Y. P., Yuan Y. F., Peng X., Song J., Liu J., Qu J. (2019). An ultrasensitive Fano resonance biosensor using two dimensional hexagonal boron nitride nanosheets: theoretical analysis. *RSC Advances*.

[6] Zheng G., Zou X., Chen Y., Xu L., Rao W. (2017). Fano resonance in graphene-MoS_2_ heterostructure-based surface plasmon resonance biosensor and its potential applications. *Optical Materials*.

[7] Ruan B., You Q., Zhu J. (2018). Fano resonance in double waveguides with graphene for ultrasensitive biosensor. *Optics Express*.

[8] Li L., Cheng C., Yang H., Ye H., Luo X., Xi M. (2020). Label-free localized surface plasmon resonance biosensor used to detect serum interleukin-10 in patients with endometrial cancer. *Acta Physica Polonica A*.

[9] Chen Y., Zhao Z. Y., Tian Y. N. (2017). Refractive index sensing mechanism of waveguide-coupled grating nanoheterostructures containing porous silicon layers. *Chinese Journal of Lasers*.

[10] Vyas H., Hegde R. S. (2020). Improved refractive-index sensing performance in medium contrast gratings by asymmetry engineering. *Optical Materials Express*.

[11] Zheng G., Zhao L., Qian L., Xian F., Xu L. (2016). Fano resonance and tunability of optical response in double-sided dielectric gratings. *Optics Communications*.

[12] Wang J., Song C., Hang J., Hu Z. D., Zhang F. (2017). Tunable Fano resonance based on grating-coupled and graphene-based Otto configuration. *Optics Express*.

[13] Wen Y., Sun Y., Deng C. (2019). High sensitivity and FOM refractive index sensing based on Fano resonance in all-grating racetrack resonators. *Optics Communications*.

[14] Chen Y., Zhou X., Zhang M., Xiao C., Ding Z., Zhou J. (2020). Fano resonance sensing based on coupled sub-wavelength dielectric grating and periodic photonic crystal. *Physics Letters A*.

[15] Lo S. C., Yeh C. W., Wang S. H. (2021). Self-referencing biosensors using Fano resonance in periodic aluminium nanostructures. *Nanoscale*.

[16] Ye Z.-B., Xu Y., Chen H., Cheng C., Han L.-J., Xiao L. (2014). A novel micro-nano structure profile control agent: graphene oxide dispersion. *Journal of Nanomaterials*.

[17] Li L. H., Hang J. C., Sun H. X., Wang L. (2017). A conjunctive multiple-criteria decision-making approach for cloud service supplier selection of manufacturing enterprise. *Advances in Mechanical Engineering*.

[18] He S., Xie W., Zhang Y. (2021). Investigation of substrate swell-induced defect formation in suspended graphene upon helium ion implantation. *Journal of Physical Chemistry C*.

[19] Wang Y., Gu J., Li X. (2022). Boosted thermal storage performance of LiOH·H2O by carbon nanotubes isolated multilayered graphene oxide frames. *Advances in Materials Science and Engineering*.

[20] Nishanth P., Vimala G., Girisha L. (2022). Study of mechanical performance of BN grafted graphene oxide hybrid aerogel for polypropylene composites. *Journal of Nanomaterials*.

[21] Li L.-H., Hang J.-C., Gao Y., Mu C.-Y. (2017). Using an integrated group decision method based on SVM, TFN-RS-AHP, and TOPSIS-CD for cloud service supplier selection. *Mathematical Problems in Engineering*.

[22] Rajamani G., Mohankumar M., Dhamodaran G., Prakash S. O., Johnson Santhosh A. (2022). Experimental studies on the performance of graphene oxide based hybrid nanopolymers for bearing applications. *International Journal of Polymer Science*.

[23] Mousavi S. M., Behbudi G., Hashemi S. A. (2021). Recent progress in electrochemical detection of human papillomavirus (HPV) via graphene-based nanosensors. *Journal of Sensors*.

[24] Li L., Mao C. (2020). Big data supported PSS evaluation decision in service-oriented manufacturing. *IEEE Access*.

[25] Lv B., Yu W., Luo J., Qian B., Asefa M. B., Li N. A. (2021). Study on the adsorption mechanism of graphene oxide by calcareous sand in south China sea. *Adsorption Science and Technology*.

[26] Li L., Mao C., Sun H., Yuan Y., Lei B. (2020). Digital twin driven green performance evaluation methodology of intelligent manufacturing: hybrid model based on fuzzy rough-sets AHP, multistage weight synthesis, and PROMETHEE II. *Complexity*.

[27] Teow Y. H., Wan M. H., Wan N. A., Mohammad A. W. (2021). Preparation of palm oil industry’s biomass-based graphene composite for the adsorptive removal of methylene blue. *Adsorption Science and Technology*.

[28] Li L., Qu T., Liu Y. (2020). Sustainability assessment of intelligent manufacturing supported by digital twin. *IEEE Access*.

[29] Tan X., Xu G., Jiang Y., Ren D. (2021). Bipolar magnetic and thermospin transport properties of graphene nanoribbons with zigzag and klein edges. *Advances in Materials Science and Engineering*.

[30] Kim Y. H., Nguyen H. Q., Park B. J., Lee H. H., Seo T. S. (2021). Characteristics of a multiple-layered graphene oxide memory thin film transistor with gold nanoparticle embedded as charging elements. *Journal of Nanomaterials*.

[31] Li L., Lei B., Mao C. (2022). Digital twin in smart manufacturing. *Journal of Industrial Information Integration*.

[32] Zhang Q., Wu L., Li J. (2022). Mechanical properties of graphene composite materials and mesonumerical experiments on the mechanical properties of unsaturated soil-rock mixtures. *Journal of Nanomaterials*.

[33] Chufa B. M., Gonfa B. A., Anshebo T. Y., Anshebo T. Y. (2022). Graphene oxide nanoadsorbent for the removal of fluoride ion from groundwater: adsorbent performance and adsorption mechanism. *Journal of Nanotechnology*.

